# Research on Location Selection Strategy for Airlines Spare Parts Central Warehouse Based on METRIC

**DOI:** 10.1155/2021/4737700

**Published:** 2021-08-18

**Authors:** Rui Wang, Yicong Qin, Hui Sun

**Affiliations:** College of Electronic Information and Automation, Civil Aviation University of China, Tianjin 300300, China

## Abstract

With the increased demands of airlines, it is important to study the location selection strategy for spare parts central warehouse in order to improve the allocation capacity of spare parts maintenance resources and reduce the operating costs of airlines. Based on the *M*/*M*/*s*/∞/∞ multiservice desk model and Multi-Echelon Technique for Recoverable Item Control (METRIC) theory, this paper proposes a spare parts supply strategy based on the spare parts pool network and establishes a location selection model for spare parts central warehouse. The particle swarm optimization (PSO) algorithm is used to iteratively optimize the location for spare parts central warehouse and adjust the location area of the central warehouse combining transportation facilities and geographical environment factors. Finally, the paper compares the operating results for multiple airlines in pooling and off-pooling states and verifies the effectiveness of the spare parts supply model and the advantages of cost control for airlines.

## 1. Introduction

The airlines spare parts are the key resources to ensure the normal operation of the airframes, on-board equipment, and ground support equipment [1]. According to the survey, the total spare parts inventory value for supporting the operations of all airlines in the global aviation market reaches US$50 billion, accounting for 75% of airline inventory funds and 25% of working capital. However, most of the airlines spare parts are redundant in fact, and only 25% of the airlines spare parts are turnover in the industry [2, 3]. With the repeated COVID-19 epidemic and the fierce competition in the aviation market, cost control has become a top priority for airlines. Therefore, how to promote the spare parts pooling among airlines to achieve a win-win situation and to reduce inventory redundancy while meeting the requirements of spare parts guarantee rate are the key to the current airlines spare parts configuration management.

Airlines spare parts configuration management is an important way to realize the reasonable airlines spare parts inventory allocation, avoid shortage or waste of airlines spare parts, improve utilization rate of airlines spare parts, ensure reliability of dispatch, and reduce operating costs [4–6]. The development of this topic originates from the Multi-Echelon Technique for Recoverable Item Control (METRIC) theory developed by the US RAND Corporation for the US Air Force. The METRIC theory is developed based on the establishment of a two-level (central warehouse level and maintenance base level) maintenance support system and optimization model. Assume that the repair capacity of repair shops is unlimited (the number of repaired equipment is unlimited), and the failure rate of parts is independent of the number of working parts [7]. Due to the long aging scrapping time of the turnover equipment in the real environment and the replacement problem of turnover parts is usually caused by the sudden failure and damage, so it is reasonable to ignore the impact of aging life [8]. This theory is widely used in the spare parts configuration management for complex equipment such as the OPUS software used by the European and American navies and air forces [9]. With the continuous development of METRIC theory, many scholars have carried out research on it from different perspectives. Aiming at the multilevel inventory problem of airlines spare parts, researchers start from the optimization problem of airlines spare parts guarantee supply inventory on the basis of the static Palm theorem and establish the METRIC model with the largest use efficiency of spare parts under the constraint of total costs [10]. On this basis, reference [11] introduces the concept of virtual inventory and improves the METRIC model with the goal of the lowest overall cost of the spare parts inventory network. Reference [12] analyzes system with METRIC theory and introduces Lagrange factors to establish a multiconstraint dynamic configuration model of aviation materials and spare parts. Subsequently, depending upon the improved model of METRIC, dynamic METRIC (DYNA-METRIC), variant of METRIC (VARI-METRIC), and a mathematical model for METRIC (MOD-METRIC) are proposed. Among them, reference [13] proposes a DYNA-METRIC model that uses an unsteady composite Poisson distribution to simulate the dynamic characteristics of the spare parts supply environment with fewer restrictions on its application. Indeed, reference [14] conducted a study to show that an exponentially distributed interarrival time becomes apparent when the number of items in a system is more than ten. Then, it can solve a series of practical engineering problems. Reference [15] employs MOD-METRIC model to optimize the total cost constraint in the weapon equipment systems and obtains the number of spare parts at each level. Reference [16] analyzes the error of the expected shortage based on the negative binomial distribution and proposes the VARI-METRIC model. Subsequently, reference [17] proposes a METRIC-based model for the optimal allocation of spare stocking problems considering uncertain demand rate and limited repair capacity at the same time. The problem of supplying spare parts for a single fleet has been studied in references [18, 19]; however, inventory allocation issue with multiairlines has not been effectively analyzed. In the context of METRIC theory, the location of the central warehouse in the system cannot be ignored. In recent years, there have been many studies on the location selection [20–23]. Reference [24] develops a decision-made analysis of spare parts logistics in emergency, determines the distribution center of disaster relief goods, and deploys vehicles for relief distribution. On the basis of economic factors, reference [25] establishes optimization model of preventive maintenance and spare parts inventory to optimize maintenance decision and inventory level. References [26, 27] establish a location strategy considering factors such as economic benefits, infrastructure conditions, natural environment traffic location conditions, policies, and regulations. References [28–31] further discuss the location problem based on special factors. These factors are divided into the following six aspects: dynamic location based on uncertain demands, location based on supply chain competition perspective, multilevel logistics center planning and location selection study, service level-based location research, location selection combining logistics demand forecasting and distribution, and location selection considering the scale of logistics center construction. A lot of studies have also carried out on the selection of optimization algorithms for airlines spare parts configuration management. References [32, 33] use genetic algorithms to optimize the delay cost caused by unexpected failures and the overall cost of airlines spare parts occupation, furthermore, analyzing the effectiveness of the method through numerical examples. Reference [34] uses particle swarm optimization (PSO) algorithm to solve the optimization problem of spare parts configuration which maximizes the airlines spare parts guarantee rate. Reference [35] builds a multiobjective optimization model and uses multiobjective ant-lion algorithm to achieve the Pareto dominance solution of airlines spare parts configuration optimization.

Although there are plenty of studies on airlines spare parts configuration management, the pooling of airlines spare parts among multiple airlines topic needs to be further focused on. The main contributions of the paper can be summarized as follows:

1. Based on METRIC theory, an airline spare parts supply strategy with the participation of multiple airlines is proposed from the airlines spare parts pooling perspective.
2. A model for the location selection of a spare parts central warehouse based on queuing theory is innovatively established to reduce the total operating cost for the multiple airlines.
3. A new PSO algorithm is developed to optimize the model along with good adaptability in terms of computational efficiency and high-dimensional model processing ability.

The rest of this paper is organized as follows.  Section 2 describes the practical problems occurred in establishing a central warehouse for airlines spares parts, and model assumptions are placed.  Section 3 proposes a location selection model for the central warehouse of airlines spare parts.  Section 4 presents a PSO algorithm model based on dynamic decreasing inertia weight.  Section 5 conducts simulations to verify the proposed model and algorithm in the previous sections. Finally, the conclusions are drawn in Section 6.

## 2. Problem Description

A number of airlines participate in coordinated deployment to realize the airlines spare parts pooling and establish an airlines spare parts central warehouse. Therefore, it is necessary to form an airlines spare parts demand network to meet all participating airlines demands. The airlines spare parts are uniformly dispatched and transported by the central warehouse, and the spare inventory of each maintenance base is reasonably allocated. If a maintenance base over the network has insufficient inventory, and Aircraft on Ground (AOG) occurred, emergency horizontal transfer among maintenance bases is carried out to minimize losses. In the end, with the goal of minimizing the total cost of airlines spare parts transportation, AOG loss, and spare parts storage cost, the location of the airlines spare parts central warehouse needs to be reasonably selected. To achieve a new pattern of alliance-based development of the airlines spare parts transfer network, the paper considers reducing ineffective competition among airlines, increasing airlines spare parts guaranteeing rate; reducing the inventory redundancy, thus reduces airline operating costs. The following assumptions are for the application consideration:

  Assumption 1: the aging life of airlines spare parts is not considered in this paper for the time being due to the long aging scrapping time of the turnover airline spare parts in the real environment.
  Assumption 2: the needs of airline spare parts always exist in each maintenance base, and the replacement demand obeys Poisson distribution. The total number of operating spare parts in the airlines spare parts pooling network is large enough; the exponential distribution can be used to approximate the interval arrival time distribution for failed items.
  Assumption 3: the supply capacity of the spare parts for central warehouse is sufficient and there is no delay in dispatching. The rate of supply support obeys the negative exponential distribution.
  Assumption 4: the transport rate and the unit cost are the constants for the same type of turnover parts.
  Assumption 5: in case of emergency horizontal transfer, the AOG time is equal to the transit time between two maintenance bases, and no other incidents occur during the transit period.

## 3. Location Selection Modeling for Central Warehouse

### 3.1. Analysis of METRIC-Based Airlines Spare Parts Supply Strategy

The replacement of spare parts at each maintenance base is subject to the first come first service (FCFS) rule, and the spare parts are replenished by a combination of direct transfer from the central warehouse and emergency horizontal transfer. As shown in Figure 1, the model of airlines spare parts replacement operation and transfer for maintenance base *i*, *i* = 1, 2,…, *n*, (hereafter abbreviated as base *i*).

In Figure 1, the dotted box represents the spare parts replacement demand waiting queue and spare parts inventory capacity of base *i*. For the spare parts replacement demand waiting queue, the priority of the replacement operations is given according to the FCFS rule. Then, replenish the spare parts inventory from the central warehouse *c* to base *i* by direct transfer. Within the direct transfer time *t*_*i*_, if the queue length *k* ≤ *s* (*k* is the total number of spare parts inventory) for base *i*, it is considered that the demand can be satisfied by the inventory of base *i* itself, and no emergency horizontal transfer is needed. If *k* > *s* within *t*_*i*_, the demand of base *i* is not able to be satisfied by its own inventory, and the emergency horizontal transfer among bases is needed to support base *i* at this time.

The optimal order quantity formula, economic order quantity (EOQ), is used to determine the direct transfer strategy from central warehouse *c* to base *i* [36].

(1) $$\begin{array}{c} Q=\sqrt{\frac{2\Omega_{i}m_{i}}{{\text{Storage}}_{c}}}, \end{array}$$

where *Q* is the optimal order quantity of airlines spare parts; *Ω*_*i*_ is the annual demand for a certain type of repairable airlines spare parts for base *i*; *m*_*i*_ is the unit transportation cost for direct transfer of spare parts from central warehouse *c* to base *i*; *Storage*_*c*_ is the annual storage cost per unit of spare parts. The (*s* − 1, *s*) inventory strategy proposed in [37] is used because of the high storage cost and the low demand of the spare parts. Obviously, the optimal order quantity, *Q*, closes to 1. Subsequently, *λ*_*i*_, the daily rate of spare parts replacement demand for base *i* as shown in equation (2), can be derived according to the average annual demand of repairable airlines spare parts model [38].

(2) $$\begin{array}{c} \lambda_{i}=\frac{T_{\text{FH}i}\cdot K\cdot N}{365\cdot T_{\text{MTBUR}}}, \end{array}$$

where *T*_FH*i*_ is the annual flight hours of a certain type of aircraft for base *i*; *K* is the average number of certain spare parts installed on the aircrafts; *N* is the fleet size of the aircraft; *T*_MTBUR_ is the mean time among unscheduled removals for the repairable spare parts. The rate of spare parts supply, *µ*_*i*_, from the central warehouse *c* to base *i* in direct transfer is shown in the following equation:

(3) $$\begin{array}{c} \mu_{i}=\frac{\bar{v}}{d_{ic}}, \end{array}$$

where *d*_*ic*_ is the distance from the central warehouse *c* to base *i*; $\bar{v}$ is the average transportation rate of this repairable spare parts. When the spare parts replacement demand of base *i* can be met by its own inventory, the spare parts inventory system at base *i* obeys the *M*/*M*/*s*/∞/∞ multiservice desk model. In this model, *μ*_*i*1_=*μ*_*i*2_=⋯=*μ*_*ik*_=*μ*_*i*_. When there is a spare parts replacement demand of queue length *k* for base *i*, the overall spare parts supply rate of the system is *kμ*_*i*_,  *k*=0,1,2,…, *s*. The supply intensity of one transfer from central warehouse *c* to base *i* is *ρ*_*i*_=*λ*_*i*_/*μ*_*i*_. The maximum supply intensity that the central warehouse *c* can provide to base *i* is *ρ*_*is*_=*λ*_*i*_/*sμ*_*i*_. To ensure the length of the queue for replacement parts not growing longer and longer, it should satisfy *ρ*_*is*_ < 1. Thus, when the demand at base *i* can be met by its own inventory, the cumulative replacement rate *C*_*i*_ (*k*) is

(4) $$\begin{array}{c} C_{i}\left(k\right)=\frac{{\left(\lambda_{i}/\mu_{i}\right)}^{k}}{k!},\;\;k=0,1,2,\ldots ,s. \end{array}$$

Therefore, *P*_*i*_(*k*) is the probability of the spare parts to be replaced at base *i* with queue length *k*.

(5) $$\begin{array}{c} P_{i}\left(k\right)=C_{i}\left(k\right)\cdot P_{i}\left(0\right)=\frac{\rho_{i}^{k}}{k!}P_{i}\left(0\right),\;k=0,1,2,\ldots ,s, \end{array}$$

where

(6) $$\begin{array}{c} P_{i}\left(0\right)={\left[\sum_{k=0}^{s-1}\frac{\rho_{i}^{k}}{k!}+\frac{\rho_{i}^{s}}{s!\left(1-\rho_{is}\right)}\right]}^{-1}. \end{array}$$

In order to meet the airline's fill rate requirements and to avoid AOG in the event of spare parts replacement operations, the following equation should be met:

(7) $$\begin{array}{c} P_{i}\left(k\leq s-1\right)=\sum_{k=0}^{s-1}P_{i}\left(k\right)\geq 98\%. \end{array}$$

When spare parts replacement demand cannot be met by its own inventory at base *i*, *i*.*e.*, the queue length *k* ≥ *s*, AOG will occur, and the exceeding portion is referred as the waiting queue. Thus, *W*_*i*_ (*s*, *ρ*_*i*_), the probability that there exists a waiting queue in base *i*, obeys the Erlang waiting formula:

(8) $$\begin{array}{c} W_{i}\left(s,\rho_{i}\right)=\overset{\infty }{\underset{k=s}{\sum }}P_{i}\left(k\right)=\frac{\rho_{i}^{s}}{s!\left(1-\rho_{is}\right)}P_{i}\left(0\right). \end{array}$$

Since the input flow of spare parts demand in the system is Poisson flow, the waiting time for replacement of spare parts at base *i*, *T*, is a continuous random variable. It satisfies the nonnegative condition and obeys negative exponential distribution on *t*_*i*_, so *T* has the Markov property. The probability of spare parts to be replaced at base *i* with *T* ≤ *t*_*i*_ is

(9) $$\begin{array}{c} P_{i}\left(T\leq t_{i}\right)=W_{i}\left(s,\rho_{i}\right)\cdot \left(1-e^{-\left(s\mu_{i}-\lambda_{i}\right)t_{i}}\right),\;t_{i}\geq 0. \end{array}$$

Then, the cumulative replacement rate, *C*_*i*_ (*k*), in the waiting queue for base *i* is

(10) $$\begin{array}{c} C_{i}\left(k\right)=\frac{{\left(\lambda_{i}/\mu_{i}\right)}^{s}}{s!}\cdot {\left(\frac{\lambda_{i}}{s\mu_{i}}\right)}^{k-s}=\frac{{\left(\lambda_{i}/\mu_{i}\right)}^{k}}{s!s^{k-s}},\;k\geq s. \end{array}$$

*P*_*i*_(*k*) is the probability that there are *k* replacement demands for spare parts at base *i* which is shown below as well:

(11) $$\begin{array}{c} P_{i}\left(k\right)=C_{i}\left(k\right)\cdot P_{i}\left(0\right)=\frac{\rho_{i}^{k}}{s!s^{k-s}}P_{i}\left(0\right),\;k\geq s. \end{array}$$

Therefore, the average waiting queue length *L*_*iq*_ is

(12) $$\begin{array}{c} L_{iq}=\frac{W_{i}\left(s,\rho_{i}\right)\cdot \rho_{is}}{1-\rho_{is}}=\overset{\infty }{\underset{k=s+1}{\sum }}\left(k-s\right)P_{i}\left(k\right)=\frac{\rho_{i}^{s}\cdot P_{i}\left(0\right)}{s!}\overset{\infty }{\underset{k=s+1}{\sum }}\left(k-s\right)\rho_{is}^{k-s}. \end{array}$$

Emergency horizontal transfer also needs to be considered when there is a waiting queue at base *i*. The transit node *j* for emergency horizontal transfer depends on the transit time *T*_*ij*_:

(13) $$\begin{array}{c} T_{ij}=\frac{d_{ij}}{\bar{v}}, \end{array}$$

where *d*_*ij*_ is the distance from base *i* to base *j*; $\bar{v}$ is the average transport rate. In addition, the transportation cost of spare parts is

(14) $$\begin{array}{c} E_{ij}=a\cdot d_{ij}, \end{array}$$

where *a* is the transportation cost of spare parts per unit distance. In case of emergency horizontal transfer, the rate of spare parts supply from base *j* to base *i* is shown in the following equation:

(15) $$\begin{array}{c} \mu_{ij}=\frac{1}{T_{ij}}. \end{array}$$

Subsequently, the spare parts supply strategy for base *i* is determined by the transit time *T*_*ij*_, as shown in Figure 2.

When there is a shortage of spare parts at base *i* to apply for emergency horizontal transfer, the node *j* corresponding to *min* (*T*_*ij*_) is selected as the supply base in preference. If base *j* is also out of stock, it is deferred to the next minimum value, etc. Since the central warehouse *c* has unlimited supply capacity, once *T*_*ij*_ ≥ *T*_*ic*_, spare parts are supplied from central warehouse *c* to base *i* by default, and other bases are not considered. According to Figure 2, it is assumed that the blue node represents the central warehouse *c* and the remaining four maintenance bases are identified as 1, 2, 3, and 4. The transit time from bases 2, 3, and 4 and central warehouse *c* to base 1 was ranked as *T*_12_ ＜ *T*_13_ ＜ *T*_1*c*_ ＜ *T*_14_. Bases 2–4 are divided into two different states according to the transit time, where the green node represents the emergency horizontal transfer node of base 1, and the red node means that the node cannot be used as the emergency horizontal transfer node of base 1. Therefore, if there is a shortage of spare parts at base 1, base 2 will make emergency horizontal transfer to base 1, and central warehouse *c* will make direct transfer to base 2 to replenish the inventory. Base 3 will provide horizontal transfer to base 1 only if base 1 generates an emergency horizontal transfer requirement and base 2 does not have inventory. Accordingly, the central warehouse *c* makes direct transfer to base 3 to replenish inventory. If bases 2 and 3 have no additional stocks simultaneously, the central warehouse *c* makes a direct transfer to base 1 to replenish the inventory. Since *T*_1*c*_ ＜ *T*_14_, base 4 does not need to provide emergency horizontal transfer to base 1. Therefore, bases 2 and 3 are called emergency horizontal transfer nodes for base 1. The priority ranking of the emergency horizontal transfer nodes for each base is shown in Table 1 according to the transfer time.

Further, the source of the actual airlines spare parts replacement demand for base 1 is shown in Figure 3, where the green node represents base 1 as an emergency horizontal transfer node for bases 2, 3, and 4.

Since *λ*_*i*_, *i* = 1, 2,…, *n*, is independent of each other and obeys Poisson distribution,

(16) $$\begin{array}{c} X∼\;P\left(\lambda \right),\\ Y∼\;P\left(\mu \right). \end{array}$$

Then, there is

(17) $$\begin{array}{c} P\left\{X=x\right\}=\frac{\lambda^{x}}{x!}e^{-\lambda },\\ P\left\{Y=y\right\}=\frac{\mu^{y}}{y!}e^{-\mu },\\ P\left\{Z=z\right\}=P\left\{X+Y=z\right\}=\overset{z}{\underset{x=0}{\sum }}P\left\{X=x\right\}\cdot P\left\{Y=z-x\right\}\\ =\overset{z}{\underset{x=0}{\sum }}\left[e^{-\lambda }\frac{\lambda^{x}}{x!}\cdot e^{-\mu }\frac{\mu^{z-x}}{\left(z-x\right)!}\right]\\ =\frac{e^{-\left(\lambda +\mu \right)}}{z!}{\left(\lambda +\mu \right)}^{z}. \end{array}$$

Any combination of variables that are independent of each other and obey the Poisson distribution still obey the Poisson distribution, that is, *Z* ~ *P*(*λ*+*μ*). Therefore, the modified combination variables are also applicable to this queuing theory model. After the formation of the airlines spare parts pooling network, the actual spare parts replacement demand rate *λ*_*r*1_ is deduced in the following equation:

(18) $$\begin{array}{c} \lambda_{r1}=\lambda_{1}+P_{2}\left(k\leq s-1\right)\cdot \lambda_{2}+P_{3}\left(k\leq s-1\right)\cdot \lambda_{3}+\left[1-P_{3}\left(k\leq s-1\right)\right]\cdot P_{4}\left(k\leq s-1\right)\cdot \lambda_{4}. \end{array}$$

Therefore, the actual spare parts replacement demand rate *λ*_*ri*_ for base *i* is

(19) $$\begin{array}{c} \lambda_{ri}=\lambda_{i}+\sum_{\theta \in \left\{I\right\}}\left\{P_{\theta }\left(k\leq s-1\right)\cdot \lambda_{\theta }\cdot \prod_{\varepsilon \in \left\{H\right\}}\left[1-P_{\varepsilon }\left(k\leq s-1\right)\right]\right\}, \end{array}$$

where *θ* is the node index which regards base *i* as an emergency horizontal transfer node; {*I*} is the set of emergency horizontal transfer nodes for *θ*; *ε* is the node with higher priority than base *i* among all the emergency horizontal transfer nodes for *θ;* {*H*} is the set of *ε*. As shown in Figure 4, the actual spare parts supply rate *µ*_*r*1_ for base 1 is a combination of *µ*_1_ and the horizontal supply rate from the emergency horizontal transfer nodes (bases 2 and 3) of base 1.

Therefore, the actual expectation of supply rate of spare parts, ${\bar{\mu }}_{ri}$, for base *i* is

(20) $$\begin{array}{c} {\bar{\mu }}_{ri}=P_{i}\left(k\leq s-1\right)\mu_{i}+\left[1-P_{i}\left(k\leq s-1\right)\right]\cdot \sum_{\tau \in \left\{V\right\}}\left\{\prod_{\sigma \in \left\{Z\right\}}\left[1-P_{\sigma }\left(k\leq s-1\right)\right]\right\}P_{\tau }\left(k\leq s-1\right)\mu_{i\tau }, \end{array}$$

where *τ* is the emergency horizontal transfer node of base *i*; {*V*} is the set of *τ*; *σ* is the base node with higher priority than *τ* among all the emergency horizontal transfer nodes of base *i*; {*Z*} is the set of *σ*; *µ*_*iτ*_ denotes the supply rate of base *τ* to base *i* for airlines spare parts.

### 3.2. The Expected Cost of Pooling Strategy on Airlines Spare Parts

The expected cost of pooling strategy on airlines spare parts consists of the expected cost of spare parts transfer, the expected cost of AOG loss, and the cost of airlines spare parts storage.

#### 3.2.1. The Expected Cost of Spare Parts Transfer

The cost of spare parts transfer is composed of the direct transfer cost if the replacement demand can be met by its own inventory and the emergency horizontal transfer cost if maintenance base cannot be met by its own inventory. The expectation cost function of spare parts transfer is shown in the following equation:

(21) $$\begin{array}{c} E_{t}=\overset{n}{\underset{i=1}{\sum }}\left\{\overset{s}{\underset{k=1}{\sum }}ad_{ic}P_{i}\left(k\right)+\sum_{\tau \in \left\{V\right\}}ad_{i\tau }P_{i}\left(k\right)\left[1-P_{i}\left(k\leq s-1\right)\right]P_{\tau }\left(k\leq s-1\right)\prod_{\sigma \in \left\{Z\right\}}\left[1-P_{\sigma }\left(k\leq s-1\right)\right]\right\}, \end{array}$$

where *d*_*ic*_ is the distance from base *i* to base *c*; *d*_*iτ*_ is the distance from base *i* to base *τ*.

#### 3.2.2. The Expected Cost of AOG Loss

The expected cost of AOG loss is shown in the following equation:.

(22) $$\begin{array}{c} E_{A}=\overset{n}{\underset{i=1}{\sum }}\underset{j\in \left\{J\right\}}{\sum }\frac{d_{ij}}{\bar{v}}\left(k-s\right)P_{i}\left(k\right)\left[1-P_{i}\left(k\leq s-1\right)\right]P_{j}\left(k\leq s-1\right)\prod_{\Omega \in \left\{N\right\}}\left[1-P_{\Omega }\left(k\leq s-1\right)\right], \end{array}$$

where *k* ≥ *s*, {*J*} is the set of horizontal transfer nodes of base *i*; {*N*} is the set of base nodes with higher priority than base *j* among all emergency horizontal transfer nodes of base *i*.

#### 3.2.3. The Storage Cost of Airlines Spare Parts

The storage cost of airlines spare parts consists of the storage cost of each node on the spare parts pooling network. The inventory capacity on each maintenance base will meet the spare parts fill rate higher than 98%. Therefore, the storage cost function of spare parts pooling is shown in the following equation:

(23) $$\begin{array}{c} E_{s}=\sum_{i=1}^{n}b\cdot s_{i}, \end{array}$$

where *b* is the unit storage cost of the spare parts; *s*_*i*_ is the inventory of spare parts at base *i*.

Therefore, the total expected cost, *E*, of the airlines spare parts pooling network is shown in the following equation:

(24) $$\begin{array}{c} E=\left(E_{t}+E_{A}\right)\cdot D+E_{s}, \end{array}$$

where *E*_*t*_ is the transfer cost of airlines spare parts per unit time consisting of both horizontal transfer costs and direct transfer costs; *E*_*A*_ is the AOG loss cost per unit time; *D* is the total time; *E*_*s*_ is the storage cost of airlines spare parts.

## 4. A New PSO Algorithm Model Based on Dynamic Decreasing Inertia Weights

### 4.1. Particle Swarm Optimization Algorithm

In the location selection model for central warehouse of the airlines spare parts pooling network, the feasible domain of the original problem is the range where mainland China is located, and the feasible solution is expressed by the latitude and longitude coordinates of the range. The paper assumes that a group of “particles” in three-dimensional space is composed of longitude, latitude, and pooling expected cost in the feasible domain, and the particle is divided into its own experienced optimal position (*p* best) and global historical optimal position (*g* best) according to the expected cost. During the (iter + 1)-th iteration, the velocity and position of the particles are updated by the following equations until the optimal solution is obtained:

(25) $$\begin{array}{c} v_{i}^{\text{iter }+\;1}=w\cdot v_{i}^{\text{iter}}+c_{1}r_{1}\left(p_{i}^{\text{iter}}-x_{i}^{\text{iter}}\right)+c_{2}r_{2}\left(p_{g}^{\text{iter}}-x_{i}^{\text{iter}}\right),\\ x_{i}^{\text{iter}+1}=x_{i}^{\text{iter}}+v_{i}^{\text{iter}+1}, \end{array}$$

where *v*_*i*_^iter^ is the velocity of particle *i* for the iter-th iteration; *P*_*i*_^iter^ is the *p* best of particle *i* for the iter-th iteration; *P*_*g*_^iter^ is the *gbest* for the iter-th iteration; *x*_*i*_^iter^ is the current position of particle *i* for the iter-th iteration; *w* is the inertia weight; *c*_1_, *c*_2_ are learning factors; *r*_1_, *r*_2_ are two mutually independent and uniformly distributed random numbers between (0, 1). In this paper, the formula for the inertia weight *w* dynamics model is shown as follows:

(26) $$\begin{array}{c} w^{\text{iter }+\;1}=w_{s}-\frac{w_{s}-w_{e}}{{\left(\text{maxgen}\right)}^{2}}{\text{iter}}^{2}, \end{array}$$

where the maximum value of the inertia weight *w*_*s*_ is taken as 0.9. The minimum value of the inertia weight *w*_*e*_ is taken as 0.4. max gen is the total number of iterations. The inertia weight *w* takes values between (0.4, 0.9). The variation of *w* along with iter is plotted, as shown in Figure 5.

In the location selection model for central warehouse, the range of feasible domains is large, and it can be seen from Figure 5 that a larger *w* value and a smaller slope at the beginning of the iteration are beneficial for the particle to perform an adequate global search, while the *w* value becomes smaller and the slope becomes larger with the increase of the number of iterations, which is beneficial for the particle to converge quickly to the global optimum.

### 4.2. Flow of the Algorithm

  Step 1: preset the scale of the particle swarm pop, the range of particle velocity, the feasible domain range of the particle, max *gen*, *w*_*s*_*w*_*e*_, *c*_1_, and *c*_2_.
  Step 2: initialize particle swarm distribution, *X* = {*x*_1_, *x*_2_,…, *x*_pop_}; set the iter as 1.
  Step 3: substitute the parameters *λ*_*ri*_ and${\bar{\mu }}_{ri}$into equations (7)–(10); update *p* best and *g* best.
  Step 4: update *w* according to the number of iterations; update the velocity *v* and position *x* of each particle according to the velocity and position update formula.
  Step 5: determine whether the number of iterations reaches max gen; if so, skip to Step 6; otherwise, let iter = iter + 1 and skip to Step 3.
  Step 6: the output *g* best is the optimal location for the central warehouse, then end.

## 5. Simulation Analysis

The paper implements a repairable airlines spare parts pooling strategy of the A320 series fleet of *A*, *B*, *C*, *D*, *E,* and *F* airlines in order to carrying out the location selection for a central warehouse of spare parts pooling network. This paper uses linear regression to fit the relationship between the flight sortie, FS, and the flight hours, FH, of airlines' A320 series fleet. Then, the paper derives the parameter, *T*_FH_, based on the annual number of FS of the A320 series fleet of all bases for an airline. The fitted relationship is shown in Figure 6.

From the fitting results, it can be concluded that the *R*-square is 0.9557 and the Adj R-square is 0.9459. Therefore, there is a good second-order linear fitting relationship between FS and FH, which is shown in the following equation:

(27) $$\begin{array}{c} \text{FH}=-79.13\cdot {\text{FS}}^{2}+3120\cdot \text{FS}+7.688\times 10^{4}. \end{array}$$

The historical database of airline *A* ∼ *F*'s A320 series aircraft fleet at each maintenance base is summarized in the VariFlight website [39] and “Statistical Data on Civil Aviation of China 2019” [40]. The airline *A* ∼ *F*'s FS at each base in China are screened, as shown in Table 2.

In airlines spare parts pooling network, *λ*_*i*_ for all maintenance bases of airlines A ∼ F on the network is calculated according to equation (2), as shown in Table 3.

Further, *µ*_*i*_ and *µ*_*ij*_ are obtained according to equations (3), (13), and (15), which are substituted into equations (19) and (20) to calculate the value of *λ*_*ri*_ and${\bar{\mu }}_{ri}$. Finally, the expectation costs are obtained by equations (21)–(24). The pooling expectation cost with the change of central warehouse location is plotted, as shown in Figure 7.

As seen in Figure 7, the lighter colors represent the higher pooling expectation cost when the location of the central warehouse *c* is chosen in that region. With the deepening of the color, the pooling expectation cost becomes lower. Therefore, it can be concluded that the existence of the optimal location within the feasible domain makes the lowest pooling expectation cost, and the more the spatial distance from the optimal location, the higher the corresponding pooling expectation cost. In turn, the pooling expectation cost model is iteratively searched for optimality according to the PSO algorithm process in Section 4.2, and the iterative results are shown in Figure 8.

Figure 8 shows that the algorithm has good convergence, and after 19 iterations of the algorithm, it can be found the lowest pooling expectation cost is with 131.4 million RMB. The final optimal location is shown with a star in Figure 9.

The red dot in Figure 9 indicates the location of the maintenance base, and the location of the red star is the optimal location of the airlines spare parts central warehouse with the lowest pooling expectation cost, whose coordinates are 113° 71′ 15.98″ E and 27° 82′ 72.61″ N. When making the plan for the location selection of the spare parts central warehouse, the lowest total cost of multiple airlines pooling should be considered but also it should be ensured that the spare parts can be quickly and efficiently transferred from the central warehouse to each base node. Therefore, on the basis of the cost optimization, locating the central warehouse on the nearby hub airport can meet the timeliness and convenience requirements of spare parts transport. According to Figure 7, the closer the spatial distance from the cost-optimal location, the lower the pooling expectation cost, so the three hub airports with the closest spatial distance to the cost-optimal location are selected, as shown in Table 4.

When considering transport facilities and geographical environment factors, all three locations can meet the logistic requirements and transportation convenience for the supply of airlines spare parts. The sum of the annual operating costs for each of the six airlines operating without a pooling strategy (i.e., off-pooling strategy) for these repairable spare parts is $267.4 million RMB.  Figure 10(a) shows that the cost savings are significantly higher with the pooling strategy mentioned in the paper than that with the off-pooling strategy.  Figure 10(b) shows the distance between the cost-optimal location and the three hub airport locations with iterations. It can be seen that as the location of the spare parts central warehouse tends to be closer to cost-optimal location, the adoption of the pooling strategy optimizes the total operating cost by about 136.25 million RMB compared to the off-pooling strategy in Figure 10(a). From Figure 10(b), it can be seen that the steady state is reached after 19 iterations, while the distance between the cost-optimal location and Changsha Huanghua International Airport is the shortest. Therefore, from the transport facilities and geographical environment factors perspective, the central warehouse of these repairable spare parts is selected to be located in the area near Changsha Huanghua International Airport, whose coordinates are 113° 23′ 82.45″ E and 28° 15′ 3.16″ N and will cost approximately 131.68 million RMB. Although the total cost rose by about 540,000 RMB associated with cost-optimal location, in fact, the convenience of spare parts transport can reduce the transport process and the transport risk and then improve the economic efficiency of the spare parts pooling alliance.

Clearly, the win-win effect of adopting multiple airlines to implement the airlines spare parts pooling strategy is significant. Finally, Figure 11 demonstrates comparison of the operational status of each indicator between the pooling and off-pooling strategies for airlines spare parts while ensuring other conditions are consistent.

It can be seen that, with the guarantee of 98% filling rate, the total inventory of spare parts required by all maintenance bases is significantly less than the off-pooling strategy when the pooling strategy is adopted, which relatively reduces the size of spare parts by 64.46% and optimizes the operation cost by 50.76%. However, the daily AOG time is higher in the pooling strategy than that in off-pooling strategy. It is because under the off-pooling strategy, the maintenance bases are supplied directly from each airline's headquarters inventory, which is generally located in the more central location of all flight routes with a shorter average direct transfer cycle. Moreover, each airline will stock large amount of inventory at each maintenance base in order to ensure the 98% fill rate. However, this approach will cause redundancy of spare parts and generate unnecessary costs. If the scale of airlines spare parts arranged in the off-pooling strategy is deployed by using the pooling strategy, it can ensure a higher fill rate of spare parts in the global environment and develop a greater scale effect. Therefore, it is meaningful to adopt pooling strategy for the overall layout of airlines spare parts.

## 6. Conclusions

This paper proposes a multiairline spare parts pooling supply strategy based on METRIC theory and establishes a central warehouse location selection model for the spare parts pooling network based on *M*/*M*/*s*/∞/∞ multiservice desk model and considers three cost factors including spare parts transfer cost, AOG loss cost, and spare parts storage cost. Subsequently, the PSO algorithm is combined with the example for model validation and simulation analysis, and the result of location selected is adjusted according to the transportation facilities and geographical environment factors around the location site. Finally, the paper compares the results of airlines operating under pooling and off-pooling strategies to verify the validity of the strategy and model. The method developed in this paper will be able to provide a theoretical basis for making effective decisions on airlines pooling and the location selection of airlines spare parts central warehouse.

## Figures and Tables

**Figure 1:** Model of airlines spare parts replacement operation and transfer for base *i.*

**Figure 2:** Spare parts supply strategy.

**Figure 3:** An example of the actual source of spare parts replacement demands for base 1.

**Figure 4:** An example of the actual source of spare parts supply for base 1.

**Figure 5:** Inertia weight varies with the number of iterations.

**Figure 6:** Linear regression between FS and FH.

**Figure 7:** The pooling expectation cost with the change of central warehouse location.

**Figure 8:** PSO algorithm iteration.

**Figure 9:** The optimal location for the airlines spare parts central warehouse.

**Figure 10:** The cost savings advantages of pooling strategy and the variation of the distance between the cost-optimal location and three hub airport locations. (a) The cost savings by adopting pooling strategy compared to the off-pooling strategy. (b) The variation of distance between the cost-optimal location and the three hub airport locations with iterations.

**Figure 11:** Comparison of the operation status of each indicator between the pooling and off-pooling strategies for airlines spare parts.

**Table 1:** The priority ranking of the emergency horizontal transfer nodes for each base.

Base number	Priority			
	Level 1	Level 2	Level 3	Level 4
1	2	3	*c*	—
2	1	3	*c*	—
3	1	2	4	*c*
4	3	1	2	*c*

**Table 2:** The FS of A320 series aircraft fleet at each base in China.

No.	City	FS
*Airline A flight schedule*		
1	Beijing	17924
2	Chengdu	28639
3	Dalian	17836
4	Fuzhou	1999
5	Guangzhou	18577
6	Guiyang	2191
7	Harbin	6085
8	Haikou	7236
9	Hangzhou	2417
10	Hefei	492
11	Kunming	13429
12	Lhasa	2959
13	Lijiang	309
14	Mianyang	4359
15	Nanchang	3129
16	Nanjing	11177
17	Ningbo	4153
18	Qingdao	2519
19	Sanya	4078
20	Shanghai	12484
21	Shenzhen	6325
22	Shenyang	9478
23	Wuxi	388
24	Wuhan	1926
25	Xi'an	2882
26	Xishuangbanna	629
27	Yinchuan	2275
28	Changchun	1753
29	Changsha	3762
30	Zhengzhou	305
31	Chongqing	16656

*Airline B flight schedule*		
1	Beihai	833
2	Chengdu	2415
3	Dalian	1982
4	Guangzhou	7132
5	Guiyang	1917
6	Guilin	1061
7	Harbin	4426
8	Hangzhou	3759
9	Hohhot	1353
10	Kunming	8356
11	Mianyang	12351
12	Nanning	3366
13	Sanya	4078
14	Shanghai	82152
15	Shenzhen	6325
16	Shenyang	6770
17	Shijiazhuang	21656
18	Urumchi	7014
19	Xi'an	4034
20	Xishuangbanna	839
21	Yinchuan	1365
22	Changchun	2103
23	Changsha	1075
24	Chongqing	4201

*Airline C flight schedule*		
1	Beihai	648
2	Beijing	50358
3	Chengdu	22773
4	Dalian	10503
5	Erdos	4711
6	Fuzhou	5998
7	Guangzhou	23553
8	Guiyang	5751
9	Guilin	909
10	Harbin	16596
11	Haikou	3515
12	Hangzhou	15305
13	Hefei	15244
14	Hohhot	2029
15	Jinan	9608
16	Kashi	343
17	Kunming	41181
18	Lhasa	1883
19	Lijiang	4332
20	Nanchang	21902
21	Nanjing	48283
22	Ningbo	14239
23	Qingdao	11336
24	Sanya	4078
25	Shanghai	117590
26	Shenzhen	22999
27	Shenyang	6319
28	Wenzhou	9870
29	Urumchi	7014
30	Wuxi	18473
31	Wuhan	2696
32	Xi'an	60516
33	Xishuangbanna	2937
34	Yinchuan	12056
35	Yulin	3265
36	Zhangjiajie	1067
37	Changchun	2454
38	Changsha	13168
39	Zhengzhou	5032
40	Chongqing	18606

*Airline D flight schedule*		
1	Beijing	40542
2	Chengdu	42786
3	Dalian	1387
4	Guangzhou	6469
5	Guiyang	7668
6	Guilin	1515
7	Harbin	6454
8	Haikou	2894
9	Hangzhou	21213
10	Kunming	6267
11	Lhasa	6994
12	Lijiang	1238
13	Mianyang	9445
14	Nanjing	3129
15	Qingdao	8817
16	Shanghai	15303
17	Shenzhen	12074
18	Shenyang	6319
19	Tianjin	2300
20	Wenzhou	8636
21	Wuxi	904
22	Wuhan	16177
23	Xi'an	11988
24	Yinchuan	5346
25	Yulin	155
26	Zhangjiajie	457
27	Changchun	1840
28	Changsha	1881
29	Zhengzhou	7928
30	Chongqing	5252

*Airline E flight schedule*		
1	Beihai	1945
2	Beijing	64014
3	Chengdu	9661
4	Dalian	28141
5	Fuzhou	2570
6	Guangzhou	74806
7	Guiyang	3834
8	Harbin	23788
9	Haikou	11577
10	Hangzhou	23361
11	Hohhot	2536
12	Jinan	8647
13	Korla	2055
14	Kunming	19099
15	Lhasa	1255
16	Lijiang	3197
17	Mianyang	5086
18	Nanchang	5811
19	Nanjing	20118
20	Nanning	3366
21	Ningbo	9493
22	Qingdao	17634
23	Sanya	12234
24	Shanghai	62017
25	Shenzhen	29324
26	Shenyang	20311
27	Tianjin	16101
28	Wenzhou	8636
29	Urumchi	4008
30	Wuxi	5038
31	Wuhan	7190
32	Xi'an	31814
33	Xishuangbanna	839
34	Yinchuan	7962
35	Yulin	3421
36	Zhangjiajie	7471
37	Changchun	15336
38	Changsha	40311
39	Zhengzhou	3202
40	Chongqing	25959

*Airline F flight schedule*		
1	Beijing	29873
2	Chengdu	28639
3	Dalian	2774
4	Fuzhou	857
5	Guangzhou	34169
6	Harbin	9036
7	Haikou	2274
8	Hangzhou	14500
9	Hefei	3442
10	Hohhot	507
11	Kunming	4178
12	Lhasa	4573
13	Lijiang	1856
14	Mianyang	10172
15	Nanchang	12515
16	Nanjing	9388
17	Nanning	3366
18	Sanya	8156
19	Shanghai	15303
20	Shenzhen	32198
21	Shenyang	25275
22	Wenzhou	8636
23	Wuxi	2713
24	Wuhan	3210
25	Xi'an	20057
26	Yinchuan	5004
27	Yulin	155
28	Changchun	2103
29	Changsha	1881
30	Zhengzhou	8081
31	Chongqing	3001

**Table 3:** *λ*_*i*_ of some bases in pooling mode.

Base *i*	Beijing	Chengdu	Dalian	Fuzhou	Guangzhou	…	Zhengzhou
*λ*_*i*_	2.361664	1.571812	0.729600	0.133096	1.918887	…	0.285990

**Table 4:** Three hub airports information with the closest spatial distance to the cost-optimal location.

Airports	Coordinates	Cost
Changsha Huanghua International Airport	(113°23′82.45″ E, 28°15′3.16″ N)	131.68 million RMB
Nanchang Changbei International Airport	(115°90′29.42″ E, 28°84′68.78″ N)	143.51 million RMB
Wuhan Tianhe International Airport	(114°25′93.49″ E, 30°81′76.41″ N)	144.98 million RMB

## Data Availability

The data used to support the findings of this study are included within the article.
